This article has been retracted.

# 3-Bromopyruvate inhibits human gastric cancer tumor growth in nude mice via the inhibition of glycolysis

**DOI:** 10.3892/ol.2014.2779

**Published:** 2014-12-08

**Authors:** SHU-LIN XIAN, WEI CAO, XIAO-DONG ZHANG, YUN-FEI LU

**Affiliations:** Department of Gastrointestinal and Gland Surgery, The First Affiliated Hospital of Guangxi Medical University, Guangxi 530021, P.R. China

**Keywords:** 3-bromopyruvate, hexokinase, nude mouse, apoptosis, treatment

## Abstract

Tumor cells primarily depend upon glycolysis in order to gain energy. Therefore, the inhibition of glycolysis may inhibit tumor growth. Our previous study demonstrated that 3-bromopyruvate (3-BrPA) inhibited gastric cancer cell proliferation *in vitro*. However, the ability of 3-BrPA to suppress tumor growth *in vivo,* and its underlying mechanism, have yet to be elucidated. The aim of the present study was to investigate the inhibitory effect of 3-BrPA in an animal model of gastric cancer. It was identified that 3-BrPA exhibited strong inhibitory effects upon xenograft tumor growth in nude mice. In addition, the antitumor function of 3-BrPA exhibited a dose-effect association, which was similar to that of the chemotherapeutic agent, 5-fluorouracil. Furthermore, 3-BrPA exhibited low toxicity in the blood, liver and kidneys of the nude mice. The present study hypothesized that the inhibitory effect of 3-BrPA is achieved through the inhibition of hexokinase activity, which leads to the downregulation of B-cell lymphoma 2 (Bcl-2) expression, the upregulation of Bcl-2-associated X protein expression and the subsequent activation of caspase-3. These data suggest that 3-BrPA may be a novel therapy for the treatment of gastric cancer.

## Introduction

Gastric cancer is a type of malignant tumor. In recent years, the prognosis of gastric cancer has improved due to the application of comprehensive treatments, in particular, surgical approaches. Despite this, the overall five-year survival rate remains low (1,2). In order to improve the clinical outcome for patients with gastric cancer, it is necessary to identify novel and effective antitumor agents.

3-Bromopyruvate (3-BrPA), a potent alkylating agent, has been identified to inhibit tumor cell proliferation by inducing cellular apoptosis (3). The induction of tumor cell apoptosis is an important mechanism to study the effectiveness of potential antitumor agents. Previous studies have confirmed that the tumor apoptotic process is regulated by apoptosis-related genes (4,5), including the anti-apoptotic B-cell lymphoma 2 (Bcl-2) gene and the pro-apoptotic Bcl-2-associated X protein (Bax) gene. By conducting studies on apoptotic gene expression, the inhibitory effect of agents on tumor growth can be analyzed. The caspase family of proteins, in which caspase-3 is the key executive molecule, play an important role in the process of apoptosis. Apoptotic stimuli activate the dimeric form of caspase-3, which is composed of hydrolyzed 17- and 12-kDa subunits. This cleaved caspase-3 is the activated form and participates in the subsequent cleavage of corresponding substrates and the induction of cellular apoptosis (6). In contrast to normal cells, tumor cells, even in the condition of sufficient oxygen, have been demonstrated to adopt glycolysis as the primary method to gain adenosine triphosphate (ATP) (7). Furthermore, ATP depletion, following the inhibition of glycolysis, has been revealed to produce persistent DNA degradation and subsequent apoptosis in tumor cells (8,9). Previous studies have identified that hexokinase (HK) is the most important enzyme in the process of glycolysis (10,11). In addition, further studies have demonstrated that 3-BrPA inhibits glycolysis by combining with the active center of HK (12–14). However, the ability of 3-BrPA to lead to tumor cell apoptosis via the inhibition of HK has yet to be elucidated.

In our previous study, it was demonstrated that 3-BrPA inhibited the proliferation of the human gastric cancer SGC-7901 cell line *in vitro* (3,15). Therefore, the aim of the present study was to identify whether 3-BrPA could suppress the growth of an implanted human gastric cancer tumor *in vivo,* and reveal the underlying mechanism.

## Materials and methods

### Reagents

The RPMI-1640 and fetal bovine serum (FBS) were purchased from HyClone Laboratories (South Logan, UT, USA). The 3-BrPA and 5-fluorouracil (5-FU) were purchased from Sigma (cat. nos. BCBD0244V and 097K1352; St. Louis, MO, USA). The UltraSensitive™ streptavidin-peroxidase (SP) immunohistochemical kit (Histostain-Plus kits; cat. no. I003-2) and HK kit were purchased from Nanjing Jiancheng Technology Co., Ltd. (cat. no. A077-1; Nanjing, China). The rabbit anti-caspase-3 (P17KD) polyclonal antibodies (1:200) were purchased from Abcam (cat. no. ab4051; Cambridge, UK). The mouse anti-human Bcl-2 monoclonal antibodies (1:200) and the secondary goat anti-mouse immunoglobulin G horseradish peroxidase (HRP)-conjugated antibodies (1:10,000) were purchased from Santa Cruz Biotechnology Inc. (cat. nos. SC-7382 and SC-2005; Santa Cruz, CA, USA). The mouse anti-human Bax monoclonal antibodies (1:5,000) were obtained from Invitrogen (cat. no. AHO0112; Carlsbad, CA, USA). The reference mouse anti-human GAPDH monoclonal antibodies (1:10,000) were purchased from Shanghai Kangcheng Biological Engineering Co., Ltd. (cat. no. KC-5G5; Shanghai, China), and the enhanced chemiluminescence (ECL) western blotting kit was obtained from Thermo Scientific (cat. no. 32109; Waltham, MA, USA).

### Cell culture and animals

The human gastric cancer SGC-7901 cell line was purchased from the cell bank of the Xiangya Medical School, Central South University (Changsha, China). The BALB/c nude mice were purchased from the animal experimental center of Guangxi Medical University (Guangxi, China). The nude mice were 5–6-week-old females, weighing between 18 and 20 g, and were fed under specific pathogen-free conditions. The experimental process was under the supervision of the Ethics Committee of Guangxi Medical University, and in accordance with internationally recognized guidelines on animal welfare.

### Proliferation assay and xenograft tumor

Following resuscitation, the SGC-7901 cells were cultured in RPMI-1640 containing 10% FBS, at 37°C in a 5% CO_2_ incubator. Cells in the logarithmic growth phase were identified and diluted with normal saline to produce a 2×10^6^/ml cell suspension. Next, the inguinal region of each mouse was subcutaneously injected with 0.2 ml cell suspension. After 10 days, xenograft tumors were produced. The animal model was successfully established once the tumor had reached a diameter of 0.5 cm. In total, 60 mice were randomly assigned to one of the following five groups (n=12): 3-BrPA high-dose group (2.67 mg/kg/day), 3-BrPA medium-dose group (2.23 mg/kg/day), 3-BrPA low-dose group (1.85 mg/kg/day), 5-FU positive control group (15 mg/kg/day) or normal saline (NS) negative control group (9,000 mg/kg/day). The 3-BrPA and 5-FU were diluted with sterile NS and injected peripherally into the tumors. Each nude mouse was injected with 0.2 ml, once per day. Continuous injections were performed for four weeks. The mice were monitored for any changes in eating, excretion or behavior. After four weeks, the mice were sacrificed by cervical dislocation.

### Transmission electron microscope (TEM) and terminal dexynucleotidyl transferase-mediated dUTP nick end labeling (TUNEL) assay

At the beginning of drug administration, and 24 h later, Vernier calipers were used to measure the tumor volume as follows: Tumor volume = ab^2^/2, where a is the long tumor diameter, and b is the short tumor diameter. The inhibition rate of the tumor volume was calculated as follows: Inhibition rate = 1 - average experimental group tumor volume/average control group tumor volume × 100. The apoptosis index (AI) was calculated by combining TUNEL and HE staining values as follows: AI = TUNEL staining positive cell numbers/tumor cell numbers × 100. The tumor specimens were observed using an H7650 TEM (Hitachi, Tokyo, Japan).

### HK activity

According to the manufacturer’s instructions in the HK kit, the experimental principle for detecting HK activity is based upon the coupling reaction with glucose-6-phosphate dehydrogenase. HK activity was measured spectrophotometrically (UV-1800; Shimadzu Corporation, Kyoto, Japan) at an absorbance of 340 nm.

### Immunohistochemistry staining (SP-assay)

The tumor specimens were collected from each group, fixed in 10% formaldehyde and then embedded in paraffin. The slides were then dewaxed using xylene and dehydrated using alcohol. Next, a 30-min incubation with 3% H_2_O_2_ was used to block endogenous peroxidase activity. Antigens were repaired using high pressure. The rabbit anti-human cleaved caspase-3 antibodies (P17KD; dilution, 1:200) were added to the slides, followed by a PBS dilution at 4°C overnight. Next, the slides were washed with PBS, and then incubated for 30 min at 37°C in a moisture chamber, prior to further washing with PBS. The slides were stained with 3,3′-diaminobenzidine, and then washed with water prior to suspension. PBS was used as a blank control to ensure reliability of the results. Each specimen was analyzed in five random visual fields under the microscope to determine tissue staining. The images were analyzed using Image-Pro Plus 6.0 software (Media Cybernetics, Warrendale, PA, USA) in order to calculate the average optical density (AOD).

### Western blot analysis

The total protein was extracted from the tumor specimens. The 10% separation gel and 5% stacking gel were prepared. A constant voltage (80 mV) was applied to seperate and stack the gel by SDS-electrophoresis for 90 min and the water bath method was used to transfer the membranes for 45 min (constant current, 100 mA). Non-specific binding was blocked using 5% skimmed milk at room temperature for 60 min. The primary antibodies against Bcl-2 (dilution, 1:2,000), Bax (dilution, 1:5,000) and GAPDH (dilution, 1:10,000) were diluted with TBST and incubated in the refrigerator at 4°C overnight. Subsequent to washing with TBST, HRP-conjugated secondary antibodies (goat anti-mouse; dilution, 1:10,000) were diluted with Tris-buffered saline with Tween 20, added to the slides and then incubated at room temperature for 1.5 h. Following further washing with TBST, ECL substrate binding was performed, exposed in a darkroom, light sheets were flushed. The grayscale values of the protein bands were determined using the Image Lab software (Bio-Rad, Hercules, CA, USA). The protein expression intensity index was based upon the ratio between gray band values and corresponding GAPDH values.

### Blood toxicity, hepatotoxicity and renal toxicity assessment

Eight blood specimens were collected from the eyeballs of each of the 12 mice in each group. Blood toxicity was evaluated by measuring the white blood cell (WBC) and platelet (PLT) counts and the hemoglobin (HGB) level. Hepatotoxicity and renal toxicity were evaluated by measuring serum alanine transaminase (ALT), albumin (ALB) and blood urea nitrogen (BUN) levels at the end of the experiment.

### Statistical analysis

The tests for each tumor specimen were repeated at least three times. The results are expressed as the mean ± standard deviation. All statistical analyses were performed using SPSS 17.0 software (SPSS, Inc., Chicago, IL, USA). Differences between multiple groups were analyzed using a one-way analysis of variance. Pairwise comparison was performed using the Student-Newman-Keuls test. A value of P<0.05 was considered to indicate a statistically significant difference.

## Results

### 3-BrPA treatment suppresses xenograft tumor growth in nude mice

During the study, no changes in eating, excretion or behavior were observed in the mice. In total, two mice succumbed to the tumor/therapy; one in the 3-BrPA high-dose group and the other in the 5-FU group. The experimental results demonstrated that xenograft tumor growth slowed, or even stopped completely, following injection with 3-BrPA or 5-FU. Furthermore, a significant difference was identified between the tumor volumes in the drug- and NS-treated groups (P<0.05). By contrast, no significant difference was identified between the tumor inhibition rates observed in the 3-BrPA high-dose- and 5-FU-treated groups (q=0.9705; P>0.05; Table I).

Following the TUNEL analysis, the AI of each group was revealed as follows: 3-BrPA high-dose group, 48.7%; 3-BrPA medium-dose group, 39.7%; 3-BrPA low-dose group, 28.7%; 5-FU group, 46.2%; and NS group, 5.1%. A significant difference was identified between the AI values of the 3-BrPA-treated groups and the NS-treated group (P<0.05). Furthermore, the results of the pairwise comparisons between the 3-BrPA groups were significantly different (P<0.05). The differences in AI between the 5-FU and 3-BrPA medium-dose groups were similar (q=1.1632; P<0.05), whereas those of the 5-FU and 3-BrPA high-dose groups were significantly different (q=5.6608; P<0.05) (Fig. 1). Upon analysis by TEM, typical features of apoptosis were observed in the 3-BrPA-treated tumors, but not in the NS-treated tumors (Fig. 2).

### 3-BrPA treatment inhibits HK activity

As shown in Table I, the HK activity observed within the 3-BrPA groups was significantly less than that in the NS group (F=178.63; P<0.01). Furthermore, HK activity decreased in a dose-dependent manner according to increasing 3-BrPA concentration. The results of the pairwise comparisons in the 3-BrPA groups were significantly different. The HK activity observed in the 5-FU group was less than that in the NS group, but more than that in the 3-BrPA low-dose group (P<0.05).

### 3-BrPA treatment suppresses expression of cleaved caspase-3

The P17KD fragment of cleaved caspase-3 was detected by immunohistochemistry. Nuclei that exhibited brown granules were considered to be positive for the expression of P17KD. The results revealed that the 5-FU-treated group had the highest positive rate of P17KD expression. The positive rate of the 3-BrPA high-dose group was less than that of the 5-FU group, but more than that of the 3-BrPA medium-dose group (F=33.806; P<0.05). No significant difference was identified between the 3-BrPA low-dose group and the 3-BrPA medium-dose or NS groups (P>0.05; Table I).

### 3-BrPA treatment suppresses expression of Bcl-2 and increases expression of Bax

The western blot analysis revealed that the expression of Bcl-2 gradually decreased with an increase in 3-BrPA dose. Expression levels in the 5-FU and 3-BrPA high-dose groups were similar (P>0.05). Each of the 3-BrPA groups demonstrated significant differences in Bcl-2 expression compared with the NS group. The expression of Bax was greater in the 3-BrPA high-dose group compared with the medium- and low-dose groups, but lower than the 5-FU group (P<0.05). The medium- and low-dose groups exhibited similar levels of Bax expression (P>0.05). Furthermore, each of the 3-BrPA groups demonstrated significant differences in the expression of Bax compared with the NS group (P<0.05; Fig. 3).

### 3-BrPA causes low blood toxicity, hepatotoxicity and renal toxicity

Overall, the WBC and PLT counts and the HGB levels in the drug-treated groups were lower than those observed in the NS group. The 5-FU group exhibited the lowest WBC, PLT and HGB levels. A significant difference was identified in the levels of WBC, PLT and HGB between the three 3-BrPA dose groups (P<0.05; Table II). Changes in the serum ALT, ALB and BUN levels, which are important indicators of liver and kidney function, were evaluated at the end of treatment. The serum ALT and BUN levels in the drug-treated groups were higher than those observed in the NS group however, the serum ALB levels in the drug-treated groups were lower than those observed in the NS group. The 5-FU group exhibited the highest ALT and BUN levels, however, the 5-FU group exhibited the lowest ALB levels. A significant difference was identified in the levels of ALT, ALB and BUN between the three 3-BrPA dose groups (P<0.05; Table III). Low levels of serum ALB and high levels of serum ALT and BUN are indicative of compromised liver function.

## Discussion

Previous studies have reported that 3-BrPA exhibits inhibitory effects upon liver cancer (16,17), breast cancer (18) and other malignant tumors (19,20). However, the ability of 3-BrPA to suppress gastric cancer growth *in vivo*, and the possible association between its inhibitory mechanism and glycolysis, remain to be elucidated. The results of the present study identified that 3-BrPA exhibits an inhibitory effect upon xenograft tumor growth in nude mice, and that the antitumor function of 3-BrPA possesses a dose-effect association, which is similar to that of the chemotherapeutic agent, 5-FU.

HK is primarily distributed throughout the mitochondria. HK is the key enzyme involved in the process of apoptosis, and is therefore associated with the rate of apoptosis. The mitochondrial membrane contains a voltage-dependent anion channel (VDAC), which when closed, can inhibit mitochondrial function. Closure of the VDAS causes changes in the permeability of the mitochondrial membrane, which following the release of proteins, such as cytochrome *c* and apoptosis factors, induces cellular apoptosis (21). HK, however, can maintain the open state of the VDAC, and therefore reduce the permeability of the mitochondrial membrane. Inhibition of HK can increase mitochondrial permeability, which leads to caspase 3 activation and the induction of apoptosis (16). A previous study revealed that 3-BrPA combines with the active region of HK, and therefore inhibits the activity of HK (22). The present study identified that the HK activity within the tumor cells from the 3-BrPA-treated groups was less than that of the cells from the 5-FU- and NS-treated groups. Furthermore, 3-BrPA dose was inversely associated with HK activity in a dose-dependent manner. This indicates that 3-BrPA can inhibit HK activity within xenograft tumor cells.

Caspase-3, also known as cysteine proteinase 32, exists in a zymogen form under normal circumstances. Caspase-3 is a key enzyme involved in mammalian cell apoptosis and is located at the center of two major apoptosis signal transduction pathways (23). Caspase-3 is involved in the inhibition of protein function, such proteins include mdm2, D4-GDI, PAK2 and PARP. The present study used immunohistochemical methods to detect the P17KD fragment of cleaved caspase-3. The results revealed that the expression of cleaved caspase-3 in the 3-BrPA-treated group was significantly higher than that in the NS group, which indicated that caspase-3 was activated by treatment with 3-BrPA. This suggests that the therapeutic action of 3-BrPA acts through the activation of caspase-3 and the subsequent initiation of cellular apoptosis.

Cellular apoptosis is an active process regulated by apoptotic genes, including Bcl-2 (24,25) and Bax (26). A member of the Bcl-2 family can be one of two types, either an inhibitor of apoptosis or a promoter of apoptosis. Bcl-2 and Bax are two important representatives. The Bcl-2 protein is able to stabilize the cellular plasma membrane, and through the inhibition of mitochondrial ion movement, can inhibit apoptosis. Therefore, Bcl-2 is considered to be one of the final common pathway members of apoptosis (26). In contrast to Bcl-2, the Bax protein promotes apoptosis. The Bcl-2 dimer regulates apoptosis by combining with Bax to form a heterodimer, which leads to the inhibition of apoptosis (27). The present study demonstrated that the expression of Bcl-2 protein in the 3-BrPA-treated groups was reduced completely. Furthermore, the reduction in the expression of Bcl-2 was associated with 3-BrPA in a dose-dependent manner. By contrast, Bax expression was significantly increased in the high- and medium-dose 3-BrPA groups, and demonstrated a gradual increase in expression according to increased 3-BrPA dose. This demonstrates that 3-BrPA can downregulate Bcl-2 expression and upregulate Bax expression in xenograft tumors, an effect that ultimately decreases the Bcl-2/Bax ratio and promotes the apoptosis of tumor cells. Overall, treatment with 3-BrPA was well tolerated, with little effect on serum WBC, PLT, HGB, ALT, ALB and BUN levels. By contrast, treatment with 5-FU increased the serum ALT and BUN levels, and decreased the WBC, PLT, HGB and ALB levels. This suggests that 3-BrPA exhibits a lower cytotoxicity upon cells compared with 5-FU. However, the potential long-term toxic effects of 3-BrPA require further investigation.

In summary, the present study identified 3-BrPA as a highly effective antitumor agent, with low cytotoxicity, for the treatment of gastric cancer. The inhibitory action of 3-BrPA may be achieved through the inhibition of HK activity, the upregulation of Bax expression, the downregulation of Bcl-2 expression and ultimately, the activation of caspase-3. 3-BrPA therefore represents a promising therapeutic strategy for the treatment of gastric cancer.

## Figures and Tables

**Figure 1:** 3-Bromopyruvate (3-BrPA) promotes tumor cell apoptosis. Images of terminal deoxynucleotidyl transferase-mediated dUTP nick end labeling revealing apoptotic tumor cells in (A) 3-BrPA high-dose, (B) 3-BrPA medium-dose, (C) 3-BrPA low-dose, (D) 5-fluorouracil (5-FU) and (E) normal saline (NS) groups (magnification, ×400). The appearance of brownish granules in the nucleus or cytoplasm is considered to represent a positive apoptotic cell. A greater proportion of positive apoptotic cells were observed in the 3-BrPA groups and the 5-FU group compared with the NS group.

**Figure 2:** Typical features of apoptosis were induced by 3-bromopyruvate (3-BrPA). Images captured by a transmission electron micropscope revealing apoptotic features in 3-BrPA medium-dose-treated tumor cells. (A) Chromatin is concentrated, (B) the shape of the nucleus is narrow and the volume is reduced, and (C) an apoptotic body is apparent. However, no typical features of apoptosis were observed in (D) normal saline-treated tumor cells.

**Figure 3:** 3-Bromopyruvate (3-BrPA) inhibits B-cell lymphoma 2 (Bcl-2) expression and promotes Bcl-2-associated X protein (Bax) expression. Representative immunoblots revealing the expression of (A) Bcl-2 and (B) Bax in the (a) NS, (b) 3-BrPA low-dose, (c) 3-BrPA medium-dose, (d) 3-BrPA high-dose and (e) 5-fluorouracil groups. Treatment with 3-BrPA decreased Bcl-2 expression and increased Bax expression in a dose-dependant manner.

**Table I:** Tumor characteristics.

Group	n	TV, mm^3^	TIR, %	HK, U/gprot	AOD
3-BrPA high-dose	11	699.9±86	45.1^a^	19.62±5.57	0.10±0.017
3-BrPA medium-dose	12	762.5±79	40.2^a^	46.26±8.68	0.07±0.009
3-BrPA low-dose	12	835.1±98	34.5^a^	67.38±13.55	0.05±0.009
5-FU	11	671.9±52	47.3^a^	103.73±8.50	0.16±0.057
NS	12	1293.8±93	-	115.81±8.45	0.04±0.008

Values are expressed as the mean ± standard deviation.

a P<0.05 vs. the NS group.

TV, tumor volume; TIR, tumor inhibition rate; HK, hexokinase; AOD, average optical density; 3-BrPA, 3-bromopyruvate; 5-FU, 5-fluorouracil; NS, normal saline.

**Table II:** WBC and PLT counts, and HGB level in each group.

Group	n	WBC, ×10^9^	PLT, ×10^9^	HGB, g/l
3-BrPA high-dose	11	2.3±0.27^a^,^b^	352±36^a^,^b^	112±6.2^a^,^b^
3-BrPA medium-dose	12	3.1±0.32^a^,^b^	371±39^a^,^b^	117±6.6^a^,^b^
3-BrPA low-dose	12	3.9±0.37^a^,^b^	412±37^b^	123±5.9^a^,^b^
5-FU	11	1.5±0.22^a^	266±32^a^	78±5.2^a^
NS	12	5.2±0.29	455±53	158±7.2

Values are expressed as the mean ± standard deviation.

a P<0.05 vs. the NS group.

b P<0.05 vs. the 5-FU group.

WBC, white blood cell; PLT, platelet; HGB, hemoglobin; 3-BrPA, 3-bromopyruvate; 5-FU, 5-fluorouracil; NS, normal saline.

**Table III:** Serum ALT, ALB and BUN levels in each group.

Group	n	ALT, mmol/l	ALB, g/l	BUN, mmol/l
3-BrPA high-dose	11	168±53^a^	59.26±2.5^a^,^b^	11.81±0.32^a^
3-BrPA medium-dose	12	152±47^a^,^b^	63.72±2.7^b^	11.22±0.45^b^
3-BrPA low-dose	12	113±38^b^	66.23±3.2^b^	10.25±0.39^b^
5-FU	11	198±56^a^	47.21±2.6^b^	12.11±0.51^a^
NS	12	102±36	68.78±2.4	9.93±0.35

Values are expressed as the mean ± standard deviation.

a P<0.05 vs. the NS group.

b P<0.05 vs. the 5-FU group.

ALT, alanine transaminase; ALB, albumin; BUN, blood urea nitrogen; 3-BrPA, 3-bromopyruvate; 5-FU, 5-fluorouracil; NS, normal saline.
